RETRACTED

# N-(1-Pyrenyl) Maleimide Induces Bak Oligomerization and Mitochondrial Dysfunction in Jurkat Cells

**DOI:** 10.1155/2015/798489

**Published:** 2015-01-08

**Authors:** Pei-Rong Huang, Shu-Chen Hung, Chia-Chu Pao, Tzu-Chien V. Wang

**Affiliations:** ^1^Department of Molecular and Cellular Biology, College of Medicine, Chang Gung University, Kwei-San, Tao-Yuan 333, Taiwan; ^2^Health Sciences Research Institute and School of Natural Sciences, University of California, Merced, CA 95343, USA; ^3^Institute of Biomedical Sciences, College of Medicine, Chang Gung University, Kwei-San, Tao-Yuan 333, Taiwan

## Abstract

N-(1-pyrenyl) maleimide (NPM) is a fluorescent reagent that is frequently used as a derivatization agent for the detection of thio-containing compounds. NPM has been shown to display a great differential cytotoxicity against hematopoietic cancer cells. In this study, the molecular mechanism by which NPM induces apoptosis was examined. Here, we show that treatment of Jurkat cells with NPM leads to Bak oligomerization, loss of mitochondrial membrane potential (Δ*ψm*), and release of cytochrome C from mitochondria to cytosol. Induction of Bak oligomerization appears to play a critical role in NPM-induced apoptosis, as downregulation of Bak by shRNA significantly prevented NPM-induced apoptosis. Inhibition of caspase 8 by Z-IETD-FMK and/or depletion of Bid did not affect NPM-induced oligomerization of Bak. Taken together, these results suggest that NPM-induced apoptosis is mediated through a pathway that is independent of caspase-8 activation.

## 1. Introduction

Apoptosis, the programmed cell death type I, plays an important role in developmental processes, maintenance of homeostasis, and elimination of damaged cells. One pathway of apoptosis is known to be triggered by the release of cytochrome C from mitochondria to cytosol, which activates the caspase cascade through the formation of a caspase-activating protein complex called the apoptosome [1, 2]. The release of cytochrome C is regulated by anti- and proapoptotic Bcl-2 family of proteins, which reside in the outer membrane of mitochondria [3]. The ratio of proapoptotic to antiapoptotic BCL-2 family proteins is a critical determinant of cytochrome C release. When the BH3-only proteins tBid and Bim are able to engage the effectors Bak and Bax, Bax and/or Bak undergoes a conformational change, leading to its oligomerization [4, 5]. The pore-forming capability of the oligomerized Bax and/or Bak results in destabilization of the mitochondrial outer membrane and subsequent release of cytochrome C from the mitochondria [6, 7].

Among the biological capabilities that are acquired during the development of human tumors, enhanced resistance to apoptosis is common in most cancers [8]. Tumor cells have evolved a variety of strategies to limit or circumvent apoptosis, including activation or enhanced expression of antiapoptotic factors (such as BCL-2, BCL-XL, and IAPs), inactivation of the master proapoptotic p53 pathway thus preventing upregulation of proapoptotic BCL-2 family proteins upon genotoxic stress [9, 10]. The induction of apoptotic cell death represents the mechanism of action for many anticancer drugs. In fact, most cytotoxic agents currently used in cancer therapy appear to exert their cytotoxic action through apoptosis induction (reviewed in [8]).

RETRACTED

During a search for anticancer drugs by screening for inhibitors of telomerase, we have identified several small molecule inhibitors, including helenalin [11] and maleimide-derived compound U-73122 [12] and N-(1-pyrenyl) maleimide (NPM) [13], that selectively inhibit telomerase in a cell-free system. One common feature of these compounds is that they are all thio-directed covalent modification agents. Although the mechanism for the selective inhibition of telomerase by these agents is presently not known, the compound NPM has been shown to display the greatest differential cytotoxicity against hematopoietic cancer cells. Surprisingly, however, through inhibition of telomerase and potentially modulation of uncharacterized targets, the primary cytotoxic effect of NPM against hematopoietic cancer cells manifests by induction of apoptosis [13]. In this study, the molecular mechanism by which NPM induces apoptosis was examined in order to advance our basic understanding for the potential application of this drug in the treatment of leukemia.

## 2. Materials and Methods

### 2.1. Chemicals, Enzymes, Antibodies, and Oligonucleotides

Fetal bovine serum (FBS), Superscript III reverse transcriptase, TRIzol reagent, and antibiotics were from Gibco-BRL.* Taq* DNA polymerase was from ABgene, Surrey, UK. Antibodies against caspases 3 (9662), 7 (9492), 8 (9746), PARP (9542), Bim (2933), Bid (2002), and Bak (6947) were purchased from Cell Signaling Technology. Antibodies against Bad (610391) and Bcl-2 (610538) were purchased from BD Biosciences. Antibody against Bcl-X_L_ (633901) was purchased from BioLegend. Anti-actin (MAB1501) antibody was purchased from Millipore. Broad-spectrum caspase inhibitor z-VAD-fmk was purchased from Promega. Caspase-8 inhibitor Z-IETD-FMK was purchased from BD Pharmingen. Gel electrophoresis reagents were from Bio-Rad. N-(1-pyrenyl) maleimide and other chemicals were from Sigma Chemical Co.

### 2.2. Cell Culture

Acute T cell leukemia-derived Jurkat (clone E6.1) cells were cultured in RPMI 1640 medium containing 10% FBS, 2 mM L-glutamine, 4.5 g/L glucose, 10 mM HEPES, 1.0 mM sodium pyruvate, and antibiotics (100 U/mL penicillin, 100 U/mL streptomycin, and 0.25 *μ*g/mL amphotericin B). Human promyelocytic leukemia HL60 cells were cultured in Iscove's modified Dulbecco's medium containing 20% FBS, 4 mM L-glutamine, and antibiotics. Human embryo kidney cells HEK293T were cultured in DMEM supplemented with 10% fetal bovine serum, 2 mM L-glutamine, and antibiotics. All cells were grown at 37°C in a humidified incubator containing 5% CO_2_.

RETRACTED

### 2.3. Measurement of Mitochondrial Membrane Potential (Δ*ψm*) Loss by Flow Cytometry

Membrane-permeable lipophilic cationic fluorochrome JC-1 (5,5′,6,6′-tetrachloro-1,1′,3,3′-tetraethylbenzimidazolcarbocyanine iodide), which exhibits potential-dependent accumulation in the mitochondria, was used to evaluate the status of Δ*ψm* according to the instruction in Flow Cytometry Mitochondrial Membrane Potential Detection Kit (BD Biosciences). In brief, 10^6^ cells were washed and resuspended in 500 *μ*L of JC-1 working solution. After incubating at 37°C for 15 min, cells were harvested and washed with Assay Buffer twice. The change in Δ*ψm* was analyzed by flow cytometry (BD FACSCalibur TM system, Becton Dickinson) using 488 nm Argon ion laser for excitation. The emitted green and red fluorescence light of JC-1 were detected by using filters 530/30 nm and 585/42 nm, respectively. Data analysis was performed with BD Cell Quest pro software (Becton Dickinson).

### 2.4. Detection of Cytochrome C Release

The release of cytochrome C from the mitochondria was assayed by FlowCellect Cytochrome C kit (Millipore). In brief, 2 × 10^5^ cells were washed and resuspended in 200 *μ*L of permeabilization buffer. After incubating on ice for 10 min, 200 *μ*L of the fixation buffer was added to each sample and incubated at room temperature for 20 min. The permeabilized cells were collected by centrifugation and then resuspended in 200 *μ*L of blocking buffer. After incubating at 25°C for 30 min, 20 *μ*L of anti-cytochrome C-FITC antibody was added to each sample and incubated at 25°C for 30 min in the dark. The cell mixture was washed with blocking buffer and a total of 10,000 cells were analyzed by flow cytometry (BD FACSCaliburTM system, Becton Dickinson) using 488 nm Argon ion laser for excitation. The emitted green (FITC) light was detected by using filters 530/30 nm. Data analysis was performed with BD Cell Quest pro software (Becton Dickinson).

### 2.5. Determination of Bak and Bax Oligomerization

*In vitro* crosslinking for the detection of Bak and Bax oligomerization was performed according to the methods of Shawgo et al. [14]. In brief, 10^6^ cells were incubated in 80 *μ*L of PBS containing 100 mM EDTA and 1 mM cross-linking agent bismaleimidohexane (BMH) at 22°C for 30 min. Following incubation, cells were quenched with 100 mM dithiothreitol for 15 min and pelleted by centrifugation. The pelleted cells were suspended in RIPA lysis buffer (25 mM Tris·HCl, pH 7.6, 150 mM NaCl, 1% NP-40, 1% sodium deoxycholate, 0.1% SDS), and the detection of Bak and Bax oligomers were assayed by Western blot.

RETRACTED

### 2.6. Plasmids

The plasmids pMD.G, pCMVdelR8.91, and pLKO.1 were purchased from National RNAi Core Facility at Academia Sinica of Taiwan. The plasmids pMD.G and pCMVdelR8.91 were used for the packaging of lentiviral particles. The plasmids that express shRNA to knock down Bak and Bid were constructed by inserting the following sequences into the lentiviral vector pLKO.1. The selected shRNA sequences for Bak and Bid were 5′-CTTCGTACCATTTTTG-3′ and 5′-TGTGTGAAAGTTTTTG-3′, respectively. The shRNA sequence 5′-TTGGCAACCGCTTTTTG-3′, which targets firefly luciferase mRNA, served as the control.

### 2.7. Lentivirus Production, Infection, and Selection of shRNA-Expressing Cells

To generate lentiviral particles, HEK293T cells were cotransfected with lentiviral plasmid and packaging plasmids (pMD.G and pCMVdelR8.91) by Arrest-In (Open Biosystems) according to manufacturer's instruction. After 16 h of transfection, media containing the transfection reagents were removed and replenished with fresh media. After incubating for another 48 h, the media containing viral particles were centrifuged at 1250 rpm for 5 min, and the supernatants were collected for the infection studies. Infection of cells with lentiviral particles was carried out at 37°C in the presence of polybrene at 8 *μ*g/mL. Cells that stably express shRNA were obtained by culturing the infected cells in the presence of puromycin at 1 *μ*g/mL for 1 week.

### 2.8. Assay for Viability

Viability of NPM-treated cells was determined by using trypan blue exclusion method and MTS assay. In brief, 10 *μ*L of cellular suspension was mixed with 10 *μ*L Trypan blue (0.05%), and the percentage of nonviable cells (stained blue) was determined by microscopic examination in a hemocytometer. MTS assay was performed according to the manufacturer's suggestions (CellTiter 96^R^ AQ_ueous_ One Solution Cell Proliferation Assay kit, Promega).

### 2.9. Western Blot

Western blot analysis was performed as previously described [15].

## 3. Results

### 3.1. NPM Induces Caspase Activation to Trigger Apoptosis

To confirm that NPM-induced cell death is associated with the activation of caspases, the kinetics of caspase activation as well as the effect of caspase inhibition on viability were analyzed in Jurkat cells. As shown in Figure 1(a), the cleavage of caspase-3, caspase-7, and PARP was readily detected as early as 3 h after exposure to 0.5 *μ*M of NPM. Pretreatment of the Jurkat cells with a broad-spectrum caspase inhibitor, z-VAD-fmk, completely inhibited the cytotoxic effect of NPM (Figure 1(b)), indicating that caspase activation plays a critical role in NPM-induced cell death.

RETRACTED

### 3.2. NPM Induces Mitochondrial Dysfunction

To determine if the apoptosis induced by NPM is mediated by activation of the mitochondrial pathway, the effects of NPM treatment on mitochondrial membrane potential (Δ*ψm*) and cytochrome C released from mitochondria were examined. For evaluation of changes in mitochondrial membrane potential (Δ*ψm*), we used a membrane permeable dye, JC-1 (5,5′,6,6′-tetrachloro-1,1′,3,3′ tetraethylbenzimidazolylcarbocyanine iodide), which exhibits potential-dependent accumulation in the mitochondria. In nonapoptotic cells with intact mitochondria, most of JC-1 exist as aggregates in the mitochondria and are detected as red fluorescence light (R1 as shown in Figure 2(a)). When the mitochondrial membrane potential collapses, the JC-1 cannot accumulate within the mitochondria and exists as monomers in the cytosol, which are detected as green fluorescence light (R2 as shown in Figure 2(a)). Therefore, loss of Δ*ψm* can be determined by the ratios of JC-1 as aggregates (R1) or as monomers (R2). As shown in Figure 2(a), when the Jurkat cells were treated with 50 *μ*M CCCP (mitochondrial membrane potential disrupter), essentially all of JC-1 was detected as monomers (R2). Quantitative analysis of Δ*ψm* as measured by the decrease of JC-1 aggregates (R1) indicated that loss of Δ*ψm* was detectable in the Jurkat cells treated with 0.5 *μ*M of NPM and was greatly increased in the cells treated with 1-2 *μ*M of NPM.

Because loss of Δ*ψm* is often associated with the release of mitochondrial intermembrane space proteins into the cytosol, we next investigated whether cytochrome C is released from the NPM-treated cells. As shown in Figure 2(b), the percentage of cells with low fluorescence (M1) increased from 6.6% in the untreated control to 17%, 75%, and 89% in the cells treated with 0.5, 1, and 2 *μ*M of NPM, indicating that cytochrome C is released from mitochondria in the cells treated with NPM.

### 3.3. NPM Induces Bak and Bax Oligomerization

Bax and Bak play a critical role in triggering mitochondria-mediated apoptosis [16, 17]. Since the Jurkat (clone E6.1) cells used in this study do not express Bax ([14] and Figure 3(a)) due to frameshift mutation resulting in premature termination of translation [18], we examined whether or not oligomerization of Bak is involved in the NPM-induced apoptosis. To address this issue, Jurkat cells were exposed to varying concentrations of NPM or 500 nM of staurosporine (as a positive control for inducing Bak oligomerization) for 3 h and then treated with membrane-permeable protein cross-linker BMH. As shown in Figure 3(b), NPM induced the formation of Bak homodimer (52 kDa), but not higher order Bak oligomers, in a concentration-dependent manner in Jurkat cells. To address if the lack of higher Bak oligomerization was unique to the Jurkat cells used in this study, we examined the induction of Bax and Bak oligomerization in HL60 cells. As shown in Figure 3(c), NPM and staurosporine induced the formation of higher oligomers of Bak and Bax in HL60 cells.

RETRACTED

### 3.4. Suppression of NPM-Induced Apoptosis by Downregulation of Bak

To clarify the role of Bak in NPM-induced apoptosis, we examined the effects of Bak depletion on NPM-induced mitochondrial dysfunction and caspase activation. Jurkat cells were infected with shRNA-expressing lentiviral particles and the cells that stably express shRNA to knock down Bak were examined for NPM-induced loss of mitochondrial membrane potential (Δ*ψm*), cytochrome C release, and caspase activation. As shown in Figure 4(a), the expression level of Bak was greatly reduced in the cells that stably express shRNA against Bak (shBak) as compared to cells that express shRNA against luciferase (shLuc). Depletion of Bak resulted in an increased resistance to NPM treatment (Figure 4(b)) and significantly suppressed the NPM-induced loss of Δ*ψm* (Figure 4(c)), cytochrome C release (Figure 4(d)), and caspase activation (Figure 4(e)), indicating that Bak plays an important role in NPM-induced apoptosis in Jurkat cells.

### 3.5. Effect of NPM on the Levels of Bcl-2 Family Members

To evaluate the role of Bcl-2 family members in governing NPM-induced release of cytochrome C from mitochondria, the expression levels of proapoptotic (Bad, Bim, Bid, and Bak) and antiapoptotic (Bcl-2, Bcl-xL and Mcl-1) Bcl-2 proteins were examined in detail. Although the level of Bcl-2 has been reported to be slightly reduced in the NPM-treated cells [13], more detailed analyses, however, have indicated that there is no significant reduction of Bcl-2 in the NPM-treated cells. As shown in Figure 5(a), the levels of Bcl-2 and two other antiapoptotic proteins, Bcl-xL and Mcl-1, were not noticeably changed in the NPM-treated cells. While the proapoptotic proteins Bad and Bak were not noticeably changed, the levels of tBid and tBim_EL_ were increased (Figure 5(b)). Kinetic analysis for the increased detection of tBid revealed that the increased tBid was readily detected in the cells treated with 0.5 *μ*M of NPM for 3 h and was accompanied with the activation of caspase 8 (Figure 5(c)). In contrast, the level of tBim_EL_ appeared to increase only at a later time (Figure 5(d)).

RETRACTED

### 3.6. Caspase-8 Activation Is Not Involved in NPM-Induced Bak Oligomerization

Since it is known that the ligation of death receptors in the extrinsic pathway can cause the activation of caspase 8 and cleavage of Bid, leading to the activation of Bak or Bax [1], we investigated whether or not activation of caspase 8 and cleavage of Bid is involved in NPM-induced oligomerization of Bak. Inhibition of caspase 8 with Z-IETD-FMK abolished the cleavage of tBid but did not affect NPM-induced oligomerization of Bak (Figure 6(a)). Depletion of Bid by shRNA greatly reduced the level of Bid, but NPM-induced Bak oligomerization was not affected (Figure 6(b)). These results suggest that activation of caspase 8 and cleavage of Bid are not involved in NPM-induced oligomerization of Bak.

## 4. Discussion

NPM is a fluorescent reagent that is frequently used as a derivatization agent for the detection of thio-containing compounds [19, 20]. While little is known about the biological effect of NPM, we have recently shown that NPM induces apoptosis and displays a great differential cytotoxicity against hematopoietic cancer cells [13], making this compound an attractive candidate to be tested for its anticancer activity* in vivo*. In this work, we demonstrated that the apoptosis induced by NPM is mediated by the activation of executioner caspases and can be fully prevented by the caspase inhibitor, z-VAD-fmk (Figure 1). NPM appears to induce apoptosis by promoting mitochondrial dysfunction in Jurkat cells, as evidenced by the loss of Δ*ψm* and the release of cytochrome C from mitochondria (Figure 2).

Activation of Bak by a conformational change has been reported in the apoptosis induced by many agents [21]. A model for Bak oligomerization has been proposed [22]. In this model, activation of Bak in the mitochondria is postulated to lead to the exposure of its BH3 domain which inserts into the hydrophobic groove of an adjacent activated Bak molecule, resulting in the formation of a symmetrical Bak homodimer. Higher oligomers of Bak may be formed by dimer-dimer interactions mediated through a cryptic interface that is exposed following Bak activation [23]. Here, we demonstrated that NPM induces the oligomerization of Bak in both Jurkat and HL-60 cells (Figure 3). Activation of Bak appears to play an important role in NPM-induced apoptosis in Jurkat cells, as downregulation of Bak increases the viability of NPM-treated cells (Figure 4(b)) and suppresses the loss of Δ*ψm* and the release of cytochrome C from mitochondria (Figures 4(c) and 4(d)).

RETRACTED

At present, the mechanism leading to the activation of Bak by NPM remains unresolved. It is known that the ligation of death receptors in the extrinsic pathway can cause the activation of caspase 8 and cleavage of Bid to tBid. The cleaved tBid induces an allosteric activation and homooligomerization of Bak, which results in destabilization of the mitochondrial outer membrane and cytochrome C efflux [1]. Although the cleavage of Bid by caspase 8 has been shown to be an important mechanism leading to the activation of Bak or Bax in the extrinsic pathway of apoptosis [24], we observed that the depletion of Bid and/or inhibition of caspase-8 by Z-IETD-FMK did not appear to affect the NPM-induced formation of Bak homodimer (Figure 6). These results suggest that NPM-induced apoptosis does not depend on the extrinsic pathway of caspase-8 activation to cleave Bid for the activation of Bak. The observed cleavage of Bid to tBid in NPM-treated cells may occur as a consequence of NPM-induced Bak oligomerization and subsequent caspase activation. In support of such a postulate, depletion of Bak effectively abolished the activation of caspase-8 by NPM (Figure 4(e)). Taken together, our results suggest that NPM-induced apoptosis is mediated through induction of Bak oligomerization by a pathway that is independent of caspase-8 activation.

## Figures and Tables

**Figure 1:** NPM-induced apoptosis in Jurkat cells is dependent on caspase activation. (a) To determine the onset of caspase activation, Jurkat cells were treated with 0.5 μM NPM for the indicated time. The cell lysates were analyzed for the cleavage of caspases 3, 7, and PARP by Western blot. Actin served as a loading control. Data shown were from a representative of three independent experiments that gave similar results. (b) Effect of caspase inhibition on the viability of NPM-treated cells. Jurkat cells were pretreated with the broad-spectrum caspase inhibitor z-VAD-fmk (50 μM) for 1 h before exposing to 0.5 μM of NPM for 24 h. Cell viability was then determined by MTS assay and trypan blue exclusion method as described in Section 2. Data shown for MTS assay are the means ± SD from four independent experiments. Data shown for trypan blue exclusion method are the means ± SD from three independent experiments.

**Figure 2:** Effect of NPM on mitochondrial dysfunction in Jurkat cells. (a) Effect of NPM on the loss of mitochondrial membrane potential (Δ*ψm*). Jurkat cells were treated with 50 μM of CCCP (mitochondrial membrane potential disrupter) or 0.5–2 μM of NPM for 3 h. The treated cells were stained with JC-1 (5,5′,6,6′-tetrachloro-1,1′,3,3′ tetraethylbenzimidazolylcarbocyanine iodide) before being analyzed for the loss of mitochondrial membrane potential (Δ*ψm*) by flow cytometry as described in Section 2. FL1-H: JC-1 green fluorescence. FL2-H: JC-1 red fluorescence. R1 and R2 are the percentage of cells with polarized Δ*ψm* and depolarized Δ*ψm*, respectively. (b) Effect of NPM on the release of cytochrome C from mitochondria to cytosol. Jurkat cells were treated with 0.5–2 μM of NPM or DMSO as control for 3 h. The treated cells were labeled with Anti-Cytochrome C-FITC antibody and analyzed by flow cytometry. FL1-H: cytochrome C-FITC. M1 and M2 are the percentage of cells with low (mitochondria that have released cytochrome C) and high (intact mitochondria) fluorescence, respectively. The M1 and M2 for the untreated cells (DMSO) are 6.6% and 93.4%, respectively. Data were from a representative of three independent experiments that gave similar results.

RETRACTED

**Figure 3:** NPM induces oligomerization of Bak and Bax. (a) Expression of Bax and Bak in Jurkat and HL60 cells. The cell lysates of Jurkat and HL60 cells were analyzed for the expression of Bax and Bak by Western blot. The effect of NPM on the oligomerization of Bak and Bax in Jurkat (b) and HL60 (c) cells was analyzed by treating the cells with NPM at 0.5–1 μM or with staurosporine (STS) at 500 nM for 3 h. The treated cells were assayed for the presence of Bax and Bak oligomers as described in Section 2. Data shown were from a representative of two independent experiments that gave similar results. Actin served as a loading control. BMH, bismaleimidohexane.

**Figure 4:** Effect of Bak knockdown on NPM-induced apoptosis in Jurkat cells. (a) Expression of Bak in the Jurkat cells that stably express shRNA against Bak (shBak) or against luciferase (shLuc). Expression of Bak in the cell lysates was assayed by Western blot. The effect of Bak knockdown on NPM-induced cytotoxicity (b), loss of mitochondrial membrane potential (Δ*ψm*) (c), the release of cytochrome C from mitochondria to cytosol (d), and caspase activation (e) were analyzed in the Jurkat cells that stably express shRNA against Bak (shBak) or against luciferase (shLuc), as described in the legends to Figures 1 and 2. Data were from a representative of three independent experiments that gave similar results.

**Figure 5:** Effect of NPM on the levels of Bcl-2 family members and caspase 8 activation in Jurkat cells. Jurkat cells were treated with 0.5–1 μM of NPM for 24 h and the cell lysates were analyzed for the levels of antiapoptotic Bcl-2 family proteins (Bcl-2, Bcl-XL, and Mcl-1) (a) and proapoptotic Bcl-2 family proteins (Bad, Bim, Bid, and Bak) (b) by Western blot. To monitor the levels of active cleaved caspase 8, tBID, and BIM over time, Jurkat cells were analyzed by Western blot ((c) and (d)). tBid, truncated Bid; Bim_EL_, Bim extra long isoform; pBim_EL_, phosphorylated Bim_EL_; tBim_EL_, truncated Bim_EL_. Bim_EL_ is one of the major isoforms produced by alternative splicing. Bim_EL_ differs from Bim_L_ by the inclusion of exon 3. Actin served as a loading control. Data were from a representative of three independent experiments that gave similar results.

RETRACTED

**Figure 6:** Effect of caspase-8 inhibition and Bid downregulation on NPM-induced Bak oligomerization. (a) Effect of caspase-8 inhibition on NPM-induced oligomerization of Bak and tBid formation. Jurkat cells were pretreated with 50 μM of caspase-8 inhibitor Z-IETD-FMK for 1 h before being exposed to 0.5 or 1 μM of NPM for 3 h. The cell lysates were then assayed for the Bak oligomers and tBid as described in Section 2. (b) Effect of Bid downregulation on NPM-induced oligomerization of Bak and tBid formation. The Jurkat cells that stably express shRNA against Bid (shBid) or against luciferase (shLuc) were treated with NPM at 0.5–1 μM for 3 h. The cell lysates of the treated cells were assayed for the Bak oligomers and tBid as described in Section 2. Data shown were from a representative of three independent experiments that gave similar results. Actin served as a loading control.
